# LncRNA HOXA10-AS functions as an oncogene by binding miR-6509-5p to upregulate Y-box binding protein 1 in gastric cancer

**DOI:** 10.1080/21655979.2022.2059615

**Published:** 2022-05-06

**Authors:** Shanshan Li, Chuanhui Lu, Xinyu Li, Fan Li, Yunfeng Zhao, Meimei Xu, Hongyu Jia, Sibo Yuan

**Affiliations:** a Department of Gastroenterology, First Hospital of Qinhuangdao, Qinhuangdao, Hebei, PR China; b Department of Colorectal Cancer Surgery, The First Affiliated Hospital of Xiamen University, School of Medicine, Xiamen University, Xiamen 361003, Fujian Province, China; c Department of Colorectal Cancer Surgery, The Third Clinical Medical College, Fujian Medical University, Fuzhou 350108, Fujian Province, China; d Department of Gastrointestinal Surgery, Quanzhou First Hospital Affiliated to Fujian Medical University, Quanzhou City 362002, Fujian Province, China; e Department of Cardiovascular Internal Medicine CCU Ward, First Hospital of Qinhuangdao, Qinhuangdao 066000, Hebei Province, China; f Department of Gastrointestinal Surgery and Xiamen City Key Laboratory of Gastrointestinal Cancer, Zhongshan Hospital, Xiamen University, Xiamen 361000, Fujian Province, China

**Keywords:** Gastric cancer, LncRNA HOXA10-AS, miR-6509-5p, Y-box binding protein 1

## Abstract

Gastric cancer (GC) is one of the serious malignant diseases, accounting for several cases globally. The prevention, discovery and cure of GC depend on its molecular mechanism. In recent decades, it has been increasingly recognized that the long noncoding RNAs (lncRNAs) have been involved in GC progression. Therefore, the present study is aimed at identifying relevant lncRNAs that could act as biomarkers for GC prognosis. LncRNA HOXA10-AS is identified to be highly expressed in GC using the ENCORI database. Kaplan-Meier plot analysis indicated that the survival rate of the patient is associated with the expression of lncRNA HOXA10-AS. Interference of HOXA10-AS inhibited GC cell proliferation, migration, and invasion as well as facilitated GC apoptosis. The targets of HOXA10-AS included miR-6509-5p and Y-box binding protein 1 (YBX1). Specifically, HOXA10-AS downregulated miR-6509-5p in GC. An increase of miR-6509-5p inhibited GC cell growth. Meanwhile, miR-6509-5p interacted with YBX1 in GC. Together, lncRNA HOXA10-AS potentially acted as an oncogene through the lncRNA HOXA10-AS/miR-6509-5p/YBX1 signaling pathway in GC.

## Highlights

- LncRNA HOXA10-AS is highly expressed in gastric cancer (GC).
- Down-regulation of HOXA10-AS inhibits tumorigenesis of GC cells *in vivo.*
- HOXA10-AS interacts with miR-6509-5p and YBX1 in GC.
- Overexpression of miR-6509-5p represses proliferation and induces apoptosis.
- LncRNA HOXA10-AS acts as an oncogene through miR-6509-5p/YBX1 in GC.

## Introduction

Gastric cancer (GC) is one of the dreadful malignancies, accounting for several cancer-based mortalities globally [1,2]. Notably, the prevention, discovery, and cure of GC stringently depend on exploring the molecular mechanism[3]. Despite the progress, it still requires more underlying mechanisms in exploring the therapeutic strategies [4,5].

Long chain non-coding ribose nucleic acids (lncRNAs), once described as ‘dark matter’ [6,7], are a kind of non-coding RNAs with a length of more than 200 nucleotides. More often, these are considered to be the by-products of RNA polymerase II with no biological functionalities [8,9]. However, as an RNA molecule in the body, lncRNAs involve in many diseases, including cancer by targeting miRNA and many biological processes, such as cell cycle, and cell differentiation [10,11]. In addition, several shreds of evidence showed that lncRNA could regulate the expression of related genes through genomic imprinting, histone modification, chromatin remodeling, transcriptional activation and inhibition, as well as nuclear transport regulation mechanisms [12,13]. Among various lncRNAs, HOXA10-AS is highly expressed in glioma and tongue cancer and can promote the occurrence and development of corresponding cancers, indicating that HOXA10-AS can participate in the occurrence and development of a variety of cancers [14,15]. Previous study found miR-6509-5p had been identified as the binding partner to interact with an lncRNASNHG6[16], affecting the proliferation, migration, and invasion abilities of hepatocellular carcinoma [14,16].

However, the expression levels and roles of the HOXA10-AS network in GC are uncertain, remaining the levels of HOXA10-AS in GC related to tumor cell-like characteristics such as abnormal proliferation, migration, and invasion of tumor cells to be revealed. HOXA10-AS has been revealed to be a bad prognostic indicator in other malignancies. Moreover, it was shown that up-regulation of HOXA10-AS favored cancer cell proliferation of lung adenocarcinoma cells. Considering these aspects, we measured the expression of HOXA10-AS in GC tissues and found it was overexpressed in GC tissues. We hypothesized HOXA10-AS could act as the oncogene in GC. Thus, we aimed to investigate the role of HOXA10-AS and its network, hopefully providing the idea for GC treatment.

To explore the therapeutic options for GC, in this study, we use quantitative reverse transcription-polymerase chain reaction (RT-qPCR) to compare the expression of HOXA10-AS in GC tissue from cancer patients and normal individuals. Then, several functional assays are performed to investigate the effect of HOXA10-AS interference in GC, such as cell viability and cell colony formation. In addition, the impact of HOXA10-AS on migration and invasive ability of GC is presented, considering that GC is prone to form distant metastases and cause recurrence and lethality. Thus we also focus on the efficacy of HOXA10-AS alteration in the inhibition of GC metastatic ability using a transwell system. Owing to the function of lncRNAs as spongers for miRNA thus, we investigate the network (the targeted miRNA and its relevant gene or protein) of HOXA10-AS and their effects on cancer proliferation, and metastasis, toward the GC treatment. Bioinformatic software and database are used to predict the network (targeted gene) of HOXA10-AS. Further, RT-qPCR analysis and dual-luciferase assay are performed to confirm the predicted results. Then, cell growth, migration, and invasion, as well as *in vivo* investigations, are performed to evaluate the roles of HOXA10-AS and its network. We believe that all the results provide novel, deeper insights into the mechanism of GC and potentially explore important therapeutic implications for GC treatment.

## Materials and methods

### Clinical specimens, cell lines, and animal model

A total number of 80 paired tissue samples containing GC tissues and correlatively adjacent normal tissues were collected under the guidelines of the Ethics committee. As per the associated protocol required, clinical tissues were snap-frozen in liquid nitrogen 60 min after surgical resection and then stored at – 80°C. This study has been approved by the research ethics committee of Zhongshan Hospital, Xiamen University, and informed consent was obtained from all the subjects.

Human gastric epithelial cell line (GES-1)and human GC cell lines (SUN-1, AGS, and HGC-27) were purchased from American Type Culture Collection (ATCC, Manassas, Virginia, USA). The cells were cultured in Roswell Park Memorial Institute formulation (RPMI)-1640 (Gibco, Grand Island, NY, USA) or Dulbecco’s modified Eagle medium (DMEM, Gibco) supplemented with 10% (v/v) fetal bovine serum (FBS, Gibco) and 1% antibiotics (100 mg/ml streptomycin and 100 U/ml penicillin). The cells were incubated in a humidified atmosphere containing 5% CO_2_ at 37°C.

Nude mice were obtained from Shanghai SLAC Laboratory Animal Co., Ltd. (Shanghai, China). All the animal protocols were approved and performed in accordance with the guidelines of the animal care and ethics committee.

### Transfection

The seeded cells were serum-starved for 4 h, and then transfection reagents were added and incubated for 48 h. The transfection for each cell type was performed by adding the lipofectamine LTX with Plus reagent (ThermoFisher Scientific, Waltham, MA, USA) that minimizes the lipofectamine cytotoxicity. Further, 50 μg of sh-RNA-plasmid or sh-NC were diluted in 500 μl of medium (Invitrogen, Carlsbad, CA, USA). The HOXA10-AS plasmid and corresponding controls were transfected into GC cells. For HOXA10-AS knockdown, the scramble control plasmid was used as a negative control. Different fragments of the lncRNA HOXA10-AS promoter were cloned into the pmirGLO vector. The negative control and miR-6509-5p mimics (GenePharma, Shanghai, China) were also transfected for 48 h.

### RNA extraction and RT-qPCR analysis

mRNA kit was used to extract the total RNA (Invitrogen). Then, the PrimeScript RT reagent kit was applied to synthesize complementary DNA (cDNA). Glyceraldehyde-3-phosphate dehydrogenase (GAPDH) and U6 were used as the internal cytoplasm and nuclear controls for mRNA. Notably, for miRNAs, cDNA was synthesized by the PrimeScript miRNA cDNA Synthesis Kit, and internal U6 was used as a control for miRNA. The primers used are listed in **Table 1**. Finally, the SYBR Premix was applied to perform RT-qPCR, and the standard 2^−ΔΔCt^ method was used to measure the relative RNA levels.

### Cell viability assay

Briefly, 5 × 10^3^ cells/well were initially seeded into a 96-well plate. After transfection and incubation, a cell counting kit (CCK)-8 kit (Invitrogen) was then used to detect cell viability. Finally, the absorbance values were measured at 450 nm in the indicated timepoints by a microplate reader (Bio-Rad, Hercules, CA, USA).

### Colony formation assay

Initially, the cells at a density of 500 cells/well were seeded into 96-well plates and incubated for 14 days. It should be noted that the medium in the wells was replenished every two days. Then, cell colonies were fixed by ethanol and stained with crystal violet. Finally, the number of cell colonies was counted using the bright field microscope.

### EdU incorporation assay

Briefly, cells with a density of 1 × 10^4^ cells/well were seeded into 96-well plates. Then, the cell proliferation after transfection was evaluated by the EdU incorporation assay kit (ThermoFisher Scientific) and detected by a fluorescence microscope (Olympus, Tokyo, Japan).

### Cell apoptosis assay

Initially, the transfected cells were collected, washed, and resuspended with the binding buffer. Then, cells were centrifuged and incubated with 100 μL of the mixture of Annexin V-FITC (5 μL) and PI (5 μL) solution (BioLegend, San Diego, CA, USA) in the dark for 20 min. Finally, the FACS Calibur system was used to examine the fluorescence intensities[17].

### Transwell assay

A total of 1 × 10^5^ cells were initially seeded on the at 8 μm pore size Transwell upper insert that precoated with (for invasion) or without 1% Matrigel gel (for migration) (Corning Life Sciences, USA). Then, 600 μL of medium supplemented with 10% FBS was filled in the lower chamber. Ethanol was used to fix the cells on the lower surface of the insert, and then 0.2% crystal violet was used to stain the cells. Finally, the cells were counted by microscope and enumerated by ImageJ software[18].

### Western blotting

RIPA lysis buffer (Beyotime, Shanghai, China) containing a protease and phosphatase inhibitor was used to extract the cell protein. Further, a Bradford assay was applied to determine the protein concentration. 20 μg of denatured protein was loaded onto 10% SDS-PAGE gels for separation. After separation, the gel was transferred to 0.22 μm NC membranes (Millipore, USA), which were immersed in specific primary antibodies solution (antibody diluted with 1:1000) after blocking. Then, the membranes were incubated with 1:2000 diluted secondary antibodies, and the protein bands were detected by an ECL system (Bio-Rad). GAPDH was used as a control.

### Tumor xenograft model and HE staining

Initially, 100 μl of PBS containing Sh-NC or Sh-HOXA10-AS transfected cells (1 × 10^7^ cells) were subcutaneously injected into female BALB/c-nu/nu mice. Then, maximum (L) and minimum (W) width were monitored, and tumor volume was calculated with the formula: V = ½LW [2]. The mice were sacrificed after 36 days, and tumors were washed and weighed. Further, the tissue morphology evaluation was characterized by Hematoxylin and eosin (H&E) staining. The animal study was approved by the research ethics committee at Zhongshan Hospital, Xiamen University.

### Immunohistochemistry staining (IHC)

Initially, the paraffin-embedded tissues were prepared for slicing, and the slides were then boiled for 90s after de-paraffinization and hydration. Subsequently, the slides were treated with H_2_O_2_ for 5 min, and a diluted ki67 antibody was applied after washing. Finally, slides were added with DAB (3, 3’-diaminobenzidine), and images were captured under an inverted microscope[19].

### Dual-luciferase assay

The dual-luciferase assay was used to confirm the binding between HOXA10-AS RNA and miR-6509-5p, miR-6509-5p, and Y-box binding protein 1 (YBX1). For the interaction of HOXA10-AS RNA and miR-6509-5p, three RNAs were synthesized according to the sequence below: a) miR-6509-5p fragment; b) the HOXA10-AS with the normal binding site; c) HOXA10-AS with the mutated binding site. Then, a and b, a and c, were sub-cloned into the luciferase reporter vector, respectively. For the binding of miR-6509-5p andYBX1, the YBX1-WT or YBX1-MUT luciferase reporter vectors and miR-6509-5p were co-transfected into GC cells. Then, AGS and SUN-1 cells were seeded in a 96-well plate and incubated overnight to allow 70% confluency. Finally, the luciferase activity was detected by a Dual-Luciferase Reporter Assay System[20].

The sequences are as follows:

HOXA10-AS WT – 5′ AACAACAGGAAACUACCUAAA 3′

miR-6509-5p – 3′ CAAGGUGACGGUGAUGGAUUA 5′

HOXA10-AS Mut – 5′ AACAACAGGAAGUCGAAGCAA 3′

YBX1 WT – 5′ GAUUGGAGCUGAAGACCUAAA 3′

miR-6509-5p – 3′ CAAGGUGACGGUGAUGGAUUA 5′

YBX1 Mut – 5′ GAUUGGAGCUGAAGGAACGUA 3′

### Statistical analysis

Data were presented as the mean ± standard deviation (S.D.). The statistical analysis was conducted by GraphPad prism. Data of different groups were compared by student’s *t*-test or analysis of variance (ANOVA) followed by Tukey test, considering the P values lesser than 0.05 as statistically significant. The association between HOXA10-AS and the prognosis of GC cancer patients was calculated with the Kaplan-Meier method. * indicates P < 0.05, ** represents P < 0.01, and *** defines P < 0.001.

## Results

### LncRNA HOXA10-AS is highly expressed in GC

Various lncRNAs are reported to be involved in cancer progression. However, the specific gene to engage in GC progression is yet to be explored. Moreover, the expression levels and roles of the lncRNA HOXA10-AS network in GC are uncertain, remaining the levels of HOXA10-AS in GC related to tumor cell-like characteristics, such as abnormal proliferation, migration, and invasion of tumor cells to be revealed. In this study, we are intended to provide novel, deeper insights into the mechanism of GC and potentially explore important therapeutic implications for GC treatment. According to ENCORI database results, it was observed that the HOXA10-AS was upregulated in GC tissues compared with normal tissues (Figure 1a). To further confirm the results, the expression levels of HOXA10-AS in GC tissues and normal tissues were detected by RT-qPCR analysis. Compared with the healthy control samples (normal tissues), HOXA10-AS showed higher expression (Figure 1b). To further evaluate the role of HOXA10-AS in GC patients’ survival rate, all GC patients are divided into HOXA10-AS-high or -low groups. As depicted in Figure 1c, patients with high HOXA10-AS presented a worse prognosis *via* Kaplan-Meier analysis compared to the high HOXA10-AS group. The expression of HOXA10-AS in the human GC cell line (Sun-1, AGS, and HGC-27) and normal epithelial cell line (GES-1) was detected by RT-qPCR analysis. It was observed that the expression levels of HOXA10-AS in GC cell lines were significantly (***P < 0.001) higher than the GES-1 cell line (Figure 1d).

**Figure 1.** **LncRNA HOXA10-AS is highly expressed in GC. A**) The expression level of HOXA10-AS in GC was analyzed by the ENCORI database. **B**) The expression levels of HOXA10-AS in 80 pairs of adjacent GC and normal tissues were detected by RT-qPCR. **C)** Kaplan-Meier curve was used to evaluate the survival time of GC patients. **D**) The expression levels of HOXA10-AS in the human GC cell lines (Sun-1, AGS, and HGC-27) and normal epithelial cell line (GES-1) were detected by RT-qPCR. * indicates P < 0.05, ** represents P < 0.01, and *** defines P < 0.001.

### Down-regulation of HOXA10-AS inhibits proliferation, migration, and invasion, as well as promotes apoptosis of GC cells

As shown in Figure 2a, compared with the corresponding control (sh-control), the expression of HOXA10-AS was significantly decreased after transfected with sh-HOXA10-AS, indicating that the sh-DNA successfully interfered with the expression of HOXA10-AS. Then, several functional assays demonstrating the proliferation, cell colony, migration, and invasion of GC cell lines were performed. The viabilities of cells at different incubation time points (0, 24, 48, and 72 h) in each group (sh-HOXA10-AS and sh-NC transfection) were detected by CCK-8 assay. Compared with the corresponding control, the interference of HOXA10-AS inhibited cell proliferation (Figure 2b). Further, the cell colony formation showed a similar trend as cell proliferation, in which the downregulation of HOXA10-AS significantly decreased the number of cell colony-forming units (Figure 2c). These results suggested that low expression of HOXA10-AS could inhibit the proliferation of GC cells. The results of the transwell cell migration and invasion experiment showed that the number of GC cells with low expression of HOXA10-AS passing through the ventricular membrane (Figure 2d) and the ventricular membrane covered with matrix EMC (Figure 2e) was significantly lesser than that in the control group. These results indicated that low expression of HOXA10-AS could inhibit the migration and invasion of GC cells. Further, the flow cytometry results showed that compared to the sh-NC group, knockdown of HOXA10-AS induced a higher apoptosis rate in both cells. It should be noted that the difference between sh-HOXA10-AS and the sh-NC group was statistically significant (figure 2f). As depicted in Figure 2g, knockdown of HOXA10-AS significantly increased the expression levels of the apoptotic proteins, Bax, cleaved caspase-3, and cleaved caspase-9, and significantly reduced the expression level of an anti-apoptotic protein Bcl-2.

**Figure 2.** **Down-regulation of HOXA10-AS inhibits proliferation, migration, and invasion, as well as promotes apoptosis of GC cells. A**) The expression levels of HOXA10-AS after transfection with sh-HOXA10-AS and sh-NC were detected by RT-qPCR. **B**) Cell proliferation in each group was detected by CCK-8 assay. **C**) Results showing the cell cloning formation (n = 3). **D**) Results of transwell cell migration assays of HOXA10-AS knockdown, and the statistical results, compared with sh-NC. **E**) Results of transwell cell invasion assays of HOXA10-AS knockdown, and the statistical results, compared with sh-NC. **F**) The percentage of apoptosis in different groups of AGS and Sun-1 cells (sh-HOXA10-AS and sh-NC) was detected by flow cytometry. **G**) The expression levels of apoptosis-related proteins in different groups of AGS and Sun-1 cells (sh-HOXA10-AS and sh-NC) were detected by Western blot. * indicates P < 0.05, ** represents P < 0.01, and *** defines P < 0.001.

### *Down-regulation of HOXA10-AS inhibits tumorigenesis of GC cells in* vivo

To further explore the *in vivo* investigations, the tumor xenograft model of nude mice was constructed. Initially, AGS and Sun-1 cells were transfected with sh-HOXA10-AS and sh-NC. Then, 1 × 10^7^ cells were inoculated into nude mice. Further, the tumor volume was monitored on day-3, 9, 15, 21, 27, 33, and 36 and enumerated using the formula, V = length x width [2] /2. From the tumor growth curve, it was observed that the sh-HOXA10-AS showed tumor inhibition effects *in vivo*. At the end of day-36, nude mice were euthanized, and tumors from different groups were isolated and weighed. As shown in Figure 3a-b, the weights of the sh-HOXA10-AS treatment group were significantly lower than the sh-NC treatment group. Finally, HE staining was used to detect the changes of tumor tissue structure, in which the tumor tissue of the sh-NC treatment group structure was clear, with dense nuclei, while, in the sh-HOXA10-AS group, the cell structure was not so tight and exhibited structural characteristics of apoptosis, such as nuclear fragmentation (Figure 3c). From Figure 3d, the Ki67 expression was decreased in the interference group. Together, we could conclude that, compared with the sh-NC group, knocking down HOXA10-AS could significantly inhibit tumor growth.

**Figure 3.** **Down-regulation of HOXA10-AS inhibits tumorigenesis of GC cells in *vivo*. A**) The tumor growth curve in nude mice. **B**) The tumor weight of mice after treatment with different groups (sh-HOXA10-AS and sh-NC). **C**) H&E staining results of different groups. **D**) Ki67 expression was detected *via* IHC in the sh-HOXA10-AS group (Scale bar = 50 μm). * indicates P < 0.05, ** represents P < 0.01, and *** defines P < 0.001.

### HOXA10-AS directly binds to and represses the expression of miR-6509-5p in GC

It was found that HOXA10-AS had multiple miR-6509-5p binding sites through the analysis of ENCORI online software (Figure 4a). Further, we figured out whether the binding site was regulated by miR-6509-5p. As shown in Figure 4b, compared with the MIC NC group, the miR-6509-5p group could significantly reduce the luciferase activity of wild-type HOXA10-AS reporter gene plasmid in the two cells, and the activity difference was significant. In the co-transfection assay of pGL3-HOXA10-AS 3'UTR WT and miR-6509-5p, or pGL3-HOXA10-AS 3'UTR WT and Mimic-NC in human AGS and Sun-1 cells, as shown in Figure 4b, compared with the MIC NC group, the miR-6509-5p group could significantly reduce the luciferase activity of wild-type HOXA10-AS reporter gene plasmid, indicating the regulation role of miR-6509-5p to the binding site. The expression level of miR-6509-5p in adjacent GC and normal tissues were compared (Figure 4c), in which the expression level of miR-6509-5p in adjacent cancer tissue was statistically higher than normal tissue. Furthermore, RT-qPCR was applied to detect the expression levels of miR-6509-5p in the human GC cell line (Sun-1, AGS, HGC-27) and normal epithelial cell line GES-1. It was revealed that in human GC cell lines (Sun-1, AGS, and HGC-27), the miR-6509-5p was highly expressed over the GES-1 (Figure 4d). In addition, RT-qPCR studies showed that the expression of miR-6509-5p increased significantly in the knockdown of the HOXA10-AS group (Figure 4e). All these data indicated that the downregulation of HOXA10-AS and the upregulation of miR-6509-5p exerted great efficacy in inhibiting tumor cell proliferation. In the meantime, the tumor cell proliferation was enhanced when the miR-6509-5p decreased, which might be resulted from the increase of HOXA10-AS.

**Figure 4.** **HOXA10-AS directly binds to and represses the expression of miR-6509-5p in GC . A**) The binding site of miR-6509-5p on HOXA10-AS was analyzed by the ENCORI database. **B**) The dual-luciferase gene reporter assay in AGS and SUN-1 cell lines. **C**) The expression level of miR-6509-5p in adjacent GC and normal tissues were detected by RT-qPCR (n = 80). **D)** The expression level of miR-6509-5p in the human GC cell lines (Sun-1, AGS, and HGC-27) and normal epithelial cell line GES-1 were detected by RT-qPCR. **E)** The expression level of miR-6509-5p in AGS and Sun-1 cells after knockdown of HOXA10-AS was detected by RT-qPCR. * indicates P < 0.05, ** represents P < 0.01, and *** defines P < 0.001.

### Overexpression of miR-6509-5p expression represses GC cell proliferation, migration, invasion and induces apoptosis

To investigate the role of miR-6509-5p in cell proliferation, initially, the AGS and Sun-1 cells were transfected with control and miR-6509-5p mimics. As shown in Figure 5a, transfection efficiency by RT-qPCR indicated that, compared with control mic, miR-6509-5p mic significantly increased the expression of miR-6509-5p. The cell viability assay with the CCK-8 kit indicated that the overexpression of miR-6509-5p inhibited cell proliferation (Figure 5b). The clonogenic ability of AGS and Sun-1 cells in different groups (control mic and miR-6509-5p MIC) was detected by clonogenic assay. As depicted in Figure 5c **and Fig. S1**, the overexpression of miR-6509-5p resulting from the miR-6509-5p mimic transfection could inhibit the number of cell colonies. Furthermore, the migration and invasion abilities of AGS and Sun-1 cells in different treatment groups were measured by transwell assay. For the migration assay, a transwell insert without Matrigel layer was used, in which the miR-6509-5p mimic transfection group showed lesser migrated cells compared with the control mimic group, indicating the overexpression of miR-6509-5p could inhibit the cell migration of AGS and Sun-1 cells (Figure 5d). In the invasive ability assessment, the insert was pre-coated with Matrigel, where the invaded cells passed through the Matrigel layer, and the insert membrane was counted. As depicted in Figure 5e, the number of invaded cells in the miR-6509-5p mimic group was significantly smaller than that of in control mimic group in both cell lines. However, in the apoptosis assay, the apoptotic cell rate in the miR-6509-5p mimic group was obviously higher than the apoptosis rate in the mimic control group. Finally, the apoptotic protein Bax, cleaved caspase-3, and cleaved caspase-9 were detected by Western blot. As depicted in Figure 5g, compared to the control mimic group, the miR-6509-5p mimic transfection group showed significantly increased expression levels of Bax, cleaved caspase-3, and cleaved caspase-9 while significantly decreasing the expression level of Bcl-2.

**Figure 5.** **Overexpression of miR-6509-5p expression represses GC cell proliferation, migration, invasion and induces apoptosis. A**) The expression of miR-6509-5p after transfection in AGS and Sun-1 cells was detected by RT-qPCR. **B)** The viabilities of AGS and Sun-1 cells with transfection were detected. **C**) The cell colony formation of AGS and Sun-1 cells in different groups was detected. **D**) The migration ability of AGS and Sun-1 cells in different groups (control mimic and miR-6509-5p mimic group) was detected by Transwell assay (without matrix EMC). **E**) The invasive ability of AGS and Sun-1 cells in different groups (control mimic and miR-6509-5p mimic group) was measured by the Transwell system. **F**) The percentage of apoptosis in different groups (control mimic and miR-6509-5p mimic group) of AGS and Sun-1 cells was detected by flow cytometry. **G)** The expression levels of apoptosis-related proteins of Bax, cleaved caspase-3, and cleaved caspase-9, as well as anti-apoptotic protein Bcl-2 in different groups of AGS and Sun-1 cells (control mimic and miR-6509-5p mimic group), were detected by Western blot. * indicates P < 0.05, ** represents P < 0.01, and *** defines P < 0.001.

### miR-6509-5p directly binds to YBX1 in GC

To figure out the network of miR-6509-5p, ENCORI online software was applied to analyze the binding ability and sites of miR-6509-5p. It was observed that miR-6509-5p possessed multiple YBX1 binding sites (Figure 6a). Then, the levels of YBX1 in GC analyzed by the database revealed that the expression of YBX1 in GC was significantly higher than in normal samples, which was further confirmed by using RT-qPCR assay (Figure 6b, c). To examine the relationship between patient survival condition and YBX1 expression, the Kaplan-Meier curve was used to evaluate the survival time of GC patients. As displayed in Figure 6d, the patients with high YBX expression showed worse patient survival. Further confirmations were made whether the miR-6509-5p would affect the expression of YBX1. The expression level of YBX1 in AGS and Sun-1 cells after knockdown of miR-6509-5p was detected by RT-qPCR. The knockdown of miR-6509-5p markedly increased the expression of YBX1 (Figure 6e). Although the quantitative RNA data indicated the negative association of miR-6509-5p with YBX1, the effect of miR-6509-5p on the YBX1 protein level was uncertain. To address this aspect, a Western blot was used to detect the protein levels of YBX1 in AGS and Sun-1 cells after miR-6509-5p mimic transfection (figure 6f). Finally, a dual-luciferase gene reporter assay was carried out in AGS and Sun-1 cells. As shown in Figure 6g, compared with mimic NC, overexpression of miR-6509-5p could inhibit luciferase activity in cells, and the inhibition was abrogated after the predicted miR-6509-5p binding site was mutated.

**Figure 6.** **miR-6509-5p directly binds to YBX1 in GC. A**) The ENCORI online software shows the multiple YBX1 binding sites of miR-6509-5p. **B**) The expression levels of YBX1 in GC were analyzed by a database. **C)** The expression levels of YBX1 in GC samples and normal samples were analyzed using RT-qPCR assay. **D**) The survival curve of patients with different YBX1 expressions. **E**) The expression levels of YBX1 in AGS and Sun-1 cells after knockdown of miR-6509-5p were detected by RT-qPCR. **F**) The expression level of YBX1 in AGS and Sun-1 cells after miR-6509-5p mimic and control mimic transfection was detected by Western blot. **G**) The dual-luciferase reporter gene experiment was carried out in AGS and Sun-1 cells. * indicates P < 0.05, ** represents P < 0.01, and *** defines P < 0.001.

### LncRNA HOXA10-AS functions as an oncogene through miR-6509-5p/YBX1 in GC

To explore the effect of the interaction of miR-6509-5p, YBX1, and sh-HOXA10-AS in GC, the miR-6509-5p inhibitor was used, along with the YBX1 plasmid sub-cloned into pcDNA. The complete experimental design included sh-NC; sh-HOXA10-AS; sh-HOXA10-AS+miR-6509-5p inhibitor; and sh-HOXA10-AS+pcDNA-YBX1 (Figure 7a, b). Then, several functional experiments were conducted. As shown in Figure 7c, the knockdown of HOXA10-AS inhibited the proliferation of cells. While cancer cell proliferation partially was increased when co-transfected with miR-6509-5p inhibitor or pcDNA-YBX1. In the cell colony formation assay, it was observed that the knockdown of HOXA10-AS could inhibit the cell colony formation, while co-transfection with miR-6509-5p inhibitor or pcDNA-YBX1 could increase the cell colony number compared to the sh-HOXA10-AS group (Figure 7d **and Fig. S2**). In terms of the migration and invasion abilities, as shown in Figure 7e, interference of HOXA10-AS decreased the migration ability of cells. However, the co-transfection with miR-6509-5p inhibitor or pcDNA-YBX1, compared to the sh-HOXA10-AS, cancer cells migration number partially increased. Similarly, the knockdown of HOXA10-AS decreased the invasive ability of cells. The invasive ability was partially increased in the case of cells co-transfected with miR-6509-5p inhibitor or pcDNA-YBX1 (figure 7f). Moreover, the knockdown of HOXA10-AS resulted in cell apoptosis, while the co-transfection with miR-6509-5p inhibitor or pcDNA-YBX1 decreased the apoptotic rate (Figure 7g).

**Figure 7.** **LncRNA HOXA10-AS functions as an oncogene through miR-6509-5p/YBX1 in GC. A**) Western blot analysis, **B**) RT-qPCR analysis exploring the interactions of miR-6509-5p, YBX1, and sh-HOXA10-AS in GC after treatment with sh-NC; sh-HOXA10-AS; sh-HOXA10-AS+miR-6509-5p inhibitor; and sh-HOXA10-AS+pcDNA-YBX1. **C**) The cell viability of AGS and Sun-1 cells were detected by the CCK-8 assay. **D**) The cell colony formation of AGS and Sun-1 cells in different groups was detected. **E**) Transwell test (without Matrigel) was used to detect the migration ability of different groups of AGS and Sun-1 cells. **F**) Transwell test (with Matrigel) was used to detect the invasion ability of different groups in AGS and Sun-1 cells. **G**) The apoptotic rates of AGS and Sun-1 cells in different groups were detected by flow cytometry. * indicates P < 0.05, ** represents P < 0.01, and *** defines P < 0.001.

## Discussion

LncRNAs are essential regulators in cancer, including oral squamous cell carcinoma (OSCC)[14]. Among various lncRNAs, HOXA10-AS was aberrantly expressed in patients with OSCC and obviously associated with prognosis in OSCC, including glioma. The upregulation of HOXA10-AS was significantly associated with glioma grade, and the interference of HOXA10-AS exerted inhibitory effects on cancer cell growth[15]. Notably, HOXA10-AS is also a bad prognostic indicator in lung adenocarcinoma tissues. In some instances, it was shown that up-regulation of HOXA10-AS in lung adenocarcinoma cells could promote cancer cell proliferation[21]. Although these investigations have confirmed its important role, HOXA10-AS role in the pathogenesis of GC is poorly understood.

In our study, ENCORI database analysis indicated that HOXA10-AS was upregulated in GC tissues compared with nontumor tissues. In addition, we identified the key functions of HOXA10-AS in cancer cell proliferation, migration, and invasion by experimental validation. In *in vitro* investigations, we used the CCK-8 kit to explore the cell viability with or without sh-HOXA10-AS transfection that would affect the expression of HOXA10-AS. The application of HOXA10-AS could significantly downregulate the expression of HOXA10-AS and thus inhibit the proliferation of GC cells. These findings were consistent with the previous studies, confirming our hypothesis that the overexpression of HOXA10-AS contributed to the pathogenesis of GC. Notably, the main reason for the high lethality of GC cancer is associated with its metastatic property. To mimic the *in vivo* metastatic behavior, we used the transwell system, in which the 8 μm pore insert with Matrigel could allow the cell migration, in which the cancer cell needed to secrete components to degrade the Matrigel and help their movement. As shown in Figure 2, the interference of HOXA10-AS, due to sh-HOXA10-AS, inhibited the cancer cell viability, colony formation, migration, and invasion as well as promoted the apoptosis and up-regulation of apoptotic protein. To further demonstrate our hypothesis, several investigations in vivo were also conducted using the xenograft nude mice as a model. Together, the results were consistent with the *in vitro* results, in which the knockdown of HOXA10-AS inhibited cancer growth and reduced tumor weight (Figure 3).

The vital roles of lncRNAs have been found to be associated with miRNA. The modulation of lncRNA on miRNA showed its effects on cell growth and metastasis, which might reflect the survival rate of GC cancer patients. In our research, we figure out the associated miRNA of HOXA10-AS, which is miR-6509-5p (Figure 4). After the RT-qPCR and a dual-luciferase assay confirmation, we were highly interested in the roles of miR-6509-5p in the proliferation and progress of GC. Thus, similar functional studies were carried out. As depicted in Figure 5, similar to the inhibitory effect on cancer cell growth from downregulation of HOXA10-AS, the overexpression of miR-6509-5p, derived from the use of miR-6509-5p mimic, prevented the metastatic behavior of both GC cancer cells. These results revealed the opposite role of HOXA10-AS and miR-6509-5p in GC cell growth.

Previous studies indicated that YBX-1, a transcription factor, could exert pro-oncogenic roles[22], promoting tumor metastasis[23], and engaging in the angiogenic switch[24]. Considering the metastatic features of GC, we analyzed the binding sites of YBX1 to miR-6509-5p. It was observed that miR-6509-5p mimic could decrease the luciferase activity of YBX1, while there was no difference between miR-6509-5p mimic and control mimic in the YBX1 mutant condition (Figure 6). Thus, we loaded the fragment of YBX1 to pcDNA vector and found that the inhibitory efficacy of sh- HOXA10-AS could be partially decreased. While the abrogated efficacy of miR-6509-5p inhibitor was a little bit higher than pcDNA- YBX1, these results showed a consistent trend in cell viability, cell colony, migration, and invasion abilities of cancer cells.

In summary, we identified the aberrant expression of HOXA10-AS in GC and found its essential pro-tumor role in cell proliferation in GC tumorigenesis. Together, these results shed new light on the mechanism and its networks for HOXA10-AS in the regulation of cell proliferation. However, some limitations were identified in this research. The in-depth network of HOXA10-AS *in vivo* must be elucidated, which we will focus on in the future. In addition, detailed functional aspects of HOXA10-AS in the soil- the tumor microenvironment are worth to be validated.

## Conclusion

In the present study, the effect of HOXA10-AS on the cell proliferation, migration, and invasion of GC cells was studied by disrupting the expression of HOXA10-AS. The effect of HOXA10-AS in cells was detected by CCK-8 assay for proliferation and cell clone formation assay. The experimental results showed that downregulation of HOXA10-AS could inhibit the proliferation of GC cells. We used a transwell system to study the effect of HOXA10-AS on migration and invasion. The results showed that interfering with the expression of HOXA10-AS could significantly inhibit the migration and invasion of GC cells, which would be beneficial for preventing the metastases of GC cancer patients. Finally, based on the results of both *in vitro* and *in vivo* analyses, we conclude that HOXA10-AS could promote GC progression by miR-6509-5p/YBX1 axis and hopefully, providing a novel potential target for GC treatment.

## Supplementary Material

Supplemental Material

## Data Availability

All the data generated and/or analyzed during this study are included in this published article.

## References

[1] Graham D, Shiotani AJG. The time to eradicate gastric cancer is now. Gut. 2005;54(6):735–738.1588877110.1136/gut.2004.056549PMC1774520

[2] Bertuccio P, Chatenoud L, Levi F, et al. Recent patterns in gastric cancer: a global overview. Int J Cancer. 2009;125(3):666–673.1938217910.1002/ijc.24290

[3] Song Z, Wu Y, Yang J, et al. Progress in the treatment of advanced gastric cancer. Tumour Bio: J Int Society Oncodevelopmental Bio Med. 2017;39(7):1010428317714626.10.1177/101042831771462628671042

[4] Fock KJAP, Therapeutics. The epidemiology and prevention of gastric cancer. Alimen Pharm Therapeutics. 2014;40(3):250–260.10.1111/apt.1281424912650

[5] Maconi G, Manes G, Porro GBJWJOGW. Role of symptoms in diagnosis and outcome of gastric cancer. World J Gastroenterology. 2008;14(8):1149.10.3748/wjg.14.1149PMC269066018300338

[6] Wu L, Liu S, Qi H, et al. Research progress on plant long non-coding RNA. Plants (Basel). 2020;9(4):408.10.3390/plants9040408PMC723799232218186

[7] Gloss BS, Dinger MEJBEBA-GRM. The specificity of long noncoding RNA expression. Biochimica et biophysica acta. 2016;1859(1):16–22.2629731510.1016/j.bbagrm.2015.08.005

[8] Xing L, Zhang X, Chen AJOL. Prognostic 4‑lncRNA‑based risk model predicts survival time of patients with head and neck squamous cell carcinoma. Oncology Letters. 2019;18(3):3304–3316.3145280910.3892/ol.2019.10670PMC6704293

[9] Ponting CP, Belgard TGJH. m. g. Transcribed dark matter: meaning or myth? Human Molecular Genetics. 2010;19(R2):R162–R168.2079810910.1093/hmg/ddq362PMC2953743

[10] Rivera C, Oliveira AK, Costa RAP, et al. Prognostic biomarkers in oral squamous cell carcinoma: a systematic review. Oral Oncology. 2017;72:38–47.2879746010.1016/j.oraloncology.2017.07.003

[11] Quinn JJ, Chang HYJNRG. Unique features of long non-coding RNA biogenesis and function. Nat Rev Genetics. 2016;17(1):47–62.2666620910.1038/nrg.2015.10

[12] Wei J-W, Huang K, Yang C, et al. Non-coding RNAs as regulators in epigenetics. Oncology Reports. 2017;37(1):3–9.2784100210.3892/or.2016.5236

[13] Statello L, Guo C-J, Chen -L-L, et al. Gene regulation by long non-coding RNAs and its biological functions. Nat Rev Molecular Cell Biology. 2021;22(2):96–118.3335398210.1038/s41580-020-00315-9PMC7754182

[14] Yan X, Cong B, Chen Q, et al. Silencing lncRNA HOXA10-AS decreases cell proliferation of oral cancer and HOXA10-antisense RNA can serve as a novel prognostic predictor. J Int Med Res. 2020;48(8):0300060520934254.10.1177/0300060520934254PMC741825832776855

[15] Dong CY, Cui J, Li DH, et al. HOXA10‑AS: a novel oncogenic long non‑coding RNA in glioma. Oncology Reports. 2018;40(5):2573–2583.3013256810.3892/or.2018.6662PMC6151881

[16] Fan X, Zhao Z, Song J, et al. LncRNA-SNHG6 promotes the progression of hepatocellular carcinoma by targeting miR-6509-5p and HIF1A. Cancer Cell Int. 2021;21(1):1–11.3366350210.1186/s12935-021-01835-wPMC7931350

[17] Pan Z, Kang X, Zeng Y, et al. A mannosylated PEI–CPP hybrid for TRAIL gene targeting delivery for colorectal cancer therapy. Chem Sci. 2017;8(35):5275–5285.28959426

[18] Kang X, Zheng Z, Liu Z, et al. Liposomal codelivery of doxorubicin and andrographolide inhibits breast cancer growth and metastasis. Molecular Pharmaceutics. 2018;15(4):1618–1626.2949886810.1021/acs.molpharmaceut.7b01164

[19] Nielsen TO, Leung SCY, Rimm DL, et al. Assessment of Ki67 in breast cancer: updated recommendations from the International Ki67 in breast cancer working group. Jnci. 2021;113(7):808–819.3336963510.1093/jnci/djaa201PMC8487652

[20] Sherf BA, Navarro SL, Hannah RR, et al. Dual-luciferase reporter assay: an advanced co-reporter technology integrating firefly and Renilla luciferase assays. Promega Notes. 1996;57(2):2–8.

[21] Ma T, Hu Y, Guo Y, et al. Tumor-Promoting Activity of Long Noncoding RNA LINC00466 in Lung Adenocarcinoma via miR-144–Regulated HOXA10 Axis. American J Pathology. 2019;189(11):2154–2170.10.1016/j.ajpath.2019.06.01431381886

[22] Ise T, Nagatani G, Imamura T, et al. Transcription factor Y-box binding protein 1 binds preferentially to cisplatin-modified DNA and interacts with proliferating cell nuclear antigen. Cancer Res. 1999;59(2):342–346.9927044

[23] Cui Y, Li F, Xie Q, et al. Disease, YBX1 mediates autophagy by targeting p110β and decreasing the sensitivity to cisplatin in NSCLC. Cell Death Disease. 2020;11(6):1–14.3256175210.1038/s41419-020-2555-4PMC7305216

[24] Ghatak S, Hascall VC, Markwald RR, et al. Folfox therapy induces feedback upregulation of cd44v6 through yb-1 to maintain stemness in colon initiating cells. Int J Molecular Sci. 2021;22(2):753.10.3390/ijms22020753PMC782864133451103

